# Clinical Efficacy, Survival, and Adverse Reaction Evaluation of Immune Checkpoint Inhibitor in Advanced Gastric Cancer: A Systematic Review and Meta-Analysis

**DOI:** 10.1155/2022/6998090

**Published:** 2022-08-23

**Authors:** Ping Zhang, Xiaomeng Zhang, Na Zhu, Feifei Zhuang, Dongmei Zhou, Ping Wang

**Affiliations:** ^1^Department of Medical Oncology, Yantaishan Hospital, Yantai 264003, China; ^2^Public Health Division, Yantaishan Hospital, Yantai 264003, China

## Abstract

**Objective:**

To systematically assess the clinical effect and survival time of immune checkpoint inhibitor (ICIs) in advanced gastric cancer (GC) and adverse reactions to provide evidence-based medicine for its enhancement and adoption.

**Methods:**

PubMed, EMBASE, ScienceDirect, Cochrane Library, China Knowledge Network database (CNKI), China VIP database, Wanfang database, and China Biomedical Literature Database (CBM) online database were searched for randomized controlled trials (RCT) of immuno-checkpoint inhibitors in advanced GC therapy. Retrieval time was limited to the period from the date the database was established to present. Separately, two researchers gathered the data. Statistical software RevMan5.4 was used to estimate bias risk according to the Cochrane Handbook 5.3 standard.

**Results:**

The computer database retrieved 1723 articles, and 465 articles were eliminated when repeated studies were removed. After screening the titles and abstracts of 287 articles, 124 articles were contained after eliminating irrelevant studies, reviews, case reports, and no control literature. After carefully reading 108 studies with insufficient data and no major outcome markers, 6 RCTs were eventually contained. 4 articles compared the levels of carcinoembryonic antigen (CEA) and carbohydrate antigen 199 (CA199) after treatment. The result indicated that the levels of serum CEA and CA199 in the study group were notably lower, and the difference was statistically significant (*P* < 0.05). The immune function indexes after treatment were compared, suggesting that the improvement of immune function indexes in the study group was notably better, and the difference was statistically significant (*P* < 0.05). Three clinical trials reported the median progression-free survival (PFS). The PFS of the study group was notably longer after treatment, and the difference was statistically significant (*P* < 0.05). The occurrence of adverse reactions after treatment was analyzed by meat, and all the literatures were analyzed. No notable differences were observed in the incidence of adverse reactions.

**Conclusion:**

ICIs associated with chemotherapy is effective when treating GC, which can effectively promote the disease control rate of patients, enhance immune function, reduce the level of tumor markers, and prolong survival time. The safety is controllable, which is worth popularizing in clinical practice. However, more studies and follow-up with higher methodological quality and longer intervention time are needed to further verify it.

## 1. Introduction

The most common malignant tumor of the digestive tract in China is gastric cancer (GC), which is highly prevalent and has a poor prognosis. GC ranked second in incidence and mortality among malignant tumors in China, right behind lung cancer, according to the results of a tumor epidemiological survey. GC is a type of malignant tumor of the digestive tract that is highly morbid and highly lethal. With the application of new treatment methods, like surgery, neoadjuvant radiotherapy, neoadjuvant chemotherapy, and targeted therapy, the treatment of GC has changed to individualized and comprehensive treatment. The short-term survival rate of patients has been improved, but the 5-year survival rate is still low [1]. East Asia is a high incidence area of GC. The morbidity and mortality of GC are high in China, especially in rural areas [2]. From clinical practice, the symptoms of early GC are often atypical with only mild epigastric discomfort, which is difficult to attract people's attention. At the time of the initial diagnosis, more than 60% of the patients had locally advanced or metastatic GC. The prognosis is often poor and the median survival time is about 1 year [3].

To treat advanced GC, the first-line treatment is platinum and 5-fluorouracil-based chemotherapy [4]. A first-line treatment for patients with GC who have HER-2 positivity has been approved for trastuzumab [5]. HER-2-positive patients with advanced first-line therapy can be treated with trastuzumab and antivascular endothelial growth factor receptor 2 antibody Amatuximab or associated with paclitaxel, while HER-2-negative patients can choose second-line therapy with docetaxel, paclitaxel, or irinotecan alone [6]. Even though chemotherapy for advanced GC patients is constantly improving and gradually diversifying, the five-year survival rate is only 20%-30% [7]. With the emergence of molecular targeted therapy and immunotherapy, especially the advent of immune checkpoint inhibitor (ICIs), the pattern of third-line therapy for advanced GC may change notably.

The antitumor mechanism of traditional chemotherapeutic drugs may regulate the immune model. In combination with PD-1, PD-L1 inhibits T cell function, inhibiting tumor immunity and promoting tumor growth. In light of the study of this mechanism, blocking the PD-1/PD-L1 signal pathway makes sense for treating patients with GC. For example, chemotherapeutic drugs such as cyclophosphamide, platinum, and paclitaxel can enhance the antigenicity of tumor cells, while paclitaxel, cisplatin, and doxorubicin enhance the sensitivity of tumor cells to immune effector cells [8, 9]. PD-1 and programmed cell death ligand 1 (PD-L1) inhibitors revolutionize the treatment of advanced solid cancer [10]. In the study of the comprehensive molecular characteristics of gastric adenocarcinoma, Min and Zhang found that the overexpression of PD-L1 was observed in 65% of GC tissues [11].

The occurrence of GC is related to unhealthy diet, Helicobacter pylori infection and Epstein-Barr virus infection. Cancerous cells evade host immune defense and attack through high expression of immune checkpoint proteins to facilitate tumor growth. ICIs block the immunosuppressive signal pathway activated by cancer cells through antibodies, to enhance the body's antitumor immunity and kill tumor cells [12, 13]. Chemotherapeutic drugs can also affect the patient's immune system, such as paclitaxel, doxorubicin, and cisplatin directly act on cytotoxic lymphocytes, paclitaxel, gemcitabine, and 5-Fu eliminate immunosuppressive cells. When immunosuppressants are used in combination with chemotherapy, in one sense, chemotherapeutic drugs enhance the patient's antitumor immune response. Antitumor immunity can be enhanced by ICIs, and subsequently, drug-resistant tumor cells can be further eradicated after chemotherapy with ICIs. In this way, ICIs may provide clinical benefits when combined with chemotherapy in antitumor therapy. Current clinical trials have also studied ICIs combined chemotherapy [14]. Based on randomized clinical trials, ICIs have shown antitumor activity and good safety when compared with chemotherapy or placebo in advanced GC. In spite of this, there exhibits no consensus on whether PD-1/PD-L1 inhibitors are successful in treating advanced GC. It is proved that the clinical efficacy of ICIs is not accurate by the effectiveness of a literature or the improvement of an evaluation index. In this context, it is very necessary to systematically, quantitatively and comprehensively analyze the results of similar independent studies through meta-analysis. This paper was to systematically assess the clinical effect and survival time of immune checkpoint inhibitor (ICIs) in advanced gastric cancer (GC) and adverse reactions to provide evidence-based medicine for its enhancement and adoption.

## 2. Research Contents and Methods

### 2.1. Sources and Retrieval Methods of Documents

Search PubMed, EMBASE, ScienceDirect, CochraneLibrary, China Journal Full-Text Database (CNKI), VIP full-text Database (VIP), Wanfang Database and Chinese Biomedical Literature data (CBM), related journals, conference papers, and degree papers were searched and collected relevant data about the use of immuno-checkpoint inhibitors when treating patients with advanced GC. Searching literatures were conducted with free words + subject words, with the key words of ICIs; GC; progression; survival time; therapeutic effect; adverse reactions; meta-analysis, from January 2010 to May 2022.

### 2.2. Inclusion and Exclusion Criteria of Literature

#### 2.2.1. Literature Inclusion Criteria

(1) Type of study: all controlled trials (CT) using immunosuppressive agents to treat patients with advanced GC. (2) Participants: all patients with advanced GC were diagnosed as GC by gastroscopy/laparoscopy. The diagnostic criteria were referred to the relevant literature [15]. The TNM stage was stage III B-IV. (3) Intervention: the study group was associated with ICIs on the basis of the control group, and the control group only received chemotherapy. Indications for the use of ICIs: there were differences in the indications of different drugs, as detailed in the relevant reference [16].

#### 2.2.2. Document Exclusion Criteria

(1) The data report was incomplete and the data could not be used; (2) the research was repeated to select the most recent studies; (3) the evaluation of the curative effect of the study was not notable.

### 2.3. Quality Evaluation and Data Extraction

1. Bias risk assessment contained in the study: for the evaluation, a bias risk assessment tool recommended by Cochrane System Review Manual 5.4 was used
2. Literature screening and data extraction: independently, two researchers screened literature, gathered data, assessed quality, and cross-checked results. A disagreement should be discussed and resolved, or a third researcher should be invited to contribute to the judgement. Note: Express document management software and Excel office software were used to manage and extract research data. If the data contained in the literature was incomplete, the author of this article would be contacted to supplement it. The content of data extraction contained (1) basic information: author, publication time, and number of cases; (2) intervention: plan, course of treatment; and (3) outcome index

### 2.4. Statistical Processing

The RevMan5.4 software originated from Cochrane collaboration network for meta-analysis. The mean and standard deviation of the net change difference of serum albumin, prealbumin, and hemoglobin in the experiment, and the control cohorts were input into RevMan5 for analysis. Because the index is a continuous variable, the weighted mean difference (WMD) is used as the effect scale, and 95% confidence interval is selected. First, *χ*^2^ test is used to determine whether there is heterogeneity between the studies, if *P* > 0.05 and *I*^2^ < 50%, it is considered that the included study is homogeneous, and the modified impact model can be collected for meta-analysis; if *P* < 0.05 and *I*^2^ ≥ 50%, when judging the homogeneity of the included study, the combined effect is needed, then choose the random effect model; if *P* < 0.05, and the source of heterogeneity could not be judged, meta-analysis was not performed, and descriptive analysis was used.

## 3. Results and Analysis

### 3.1. The Results of Literature Retrieval and the Basic Situation of Literature Inclusion

The computer database retrieved 1723 articles, and 465 articles were eliminated when repeated studies were removed. After screening the titles and abstracts of 287 articles, 124 articles were contained after eliminating irrelevant studies, reviews, case reports, and no control literature. After carefully reading 108 studies with insufficient data and no major outcome markers, 6 RCTs were eventually contained [15–21]. The meta-analysis covered 492 samples in total. Illustration of literature screening was shown in Figure 1. Basic characteristics of literature was shown in Table 1.

### 3.2. Evaluation of the Quality of the Methodology Contained in the Literature

The six CT articles contained in this meta-analysis reported the baseline health status of the patients. The six studies contained all gave detailed intervention measures and treatment time. None of the 6 articles described in detail the number and reasons of the blind method and those who lost follow-up or withdrew. According to the Jadad scale, all the 6 articles were less than 2 points (Figures 2 and 3).

### 3.3. Results of Meta-Analysis

#### 3.3.1. Disease Control Rate

There were 492 samples from 6 studies contained in this study. The disease control rates were analyzed by meta. The results of heterogeneity test indicated that the research data contained in the study showed distinct heterogeneity. Chi^2^ = 5.46, df = 4, *P* = 0.24, and *I*^2^ = 27%, without obvious heterogeneity among the contained data. The analysis of random effect model (Figure 4) indicated that the disease control rate of the study group was notably better, and the difference was statistically significant (*P* < 0.05). It is suggested that the use of ICIs when treating patients with advanced GC can notably enhance the disease control rate.

#### 3.3.2. Levels of Serum Tumor Markers

Four of them compared the levels of CEA and CA199 after treatment. The results of heterogeneity test indicated that: CEA: chi^2^ = 76.60, df = 2, *P* < 0.00001, *I*^2^ = 97%; CA199: chi^2^ = 72.37, df = 2, *P* < 0.00001, *I*^2^ = 97%. Based on the summary analysis of all the literatures, the heterogeneity test results indicated that chi^2^ = 278.10, df = 5, *P* < 0.00001, *I*^2^ = 98%, indicating that the research data contained in the study showed distinct heterogeneity. The analysis of random effect model (Figure 5) indicated that the levels of serum CEA and CA199 in the study group were notably lower after treatment, and the difference was statistically significant (*P* < 0.05). It has suggested that the treatment of patients with advanced GC with ICIs can better inhibit tumor progression and alleviate the disease.

#### 3.3.3. Immune Function Index Level

There were 492 samples from 6 studies contained in this study. The immune function indexes after treatment were compared. The results of heterogeneity test indicated that CD3+: chi^2^ = 45.60, df = 1, *P* < 0.00001, *I*^2^ = 98%; CD4+: chi^2^ = 112.66, df = 2, *P* < 0.00001, *I*^2^ = 98%; CD8+: chi^2^ = 34.93, df = 2, *P* < 0.00001, *I*^2^ = 94%. It indicated that the research data contained in the study showed distinct heterogeneity. The analysis of random effect model (Figure 6) indicated that the improvement of immune function indexes in the study group was notably better after treatment, and the difference was statistically significant (*P* < 0.05). It has suggested that ICIs therapy can protect and enhance the immune function and reshape the antitumor immune system.

#### 3.3.4. Survival Period

This study contained 6 studies with a total of 492 samples, of which 3 clinical trials reported postoperative median PFS. The results of heterogeneity test indicated that the research data contained in the study showed distinct heterogeneity (chi^2^ = 17.29, df = 2, *P* = 0.0002, *I*^2^ = 88%). The analysis of random effect model (Figure 7) indicated that the PFS of the study group was notably longer after treatment, and the difference was statistically significant (*P* < 0.05). It has suggested that immuno-checkpoint inhibitor therapy can notably prolong the survival time of patients with advanced GC.

#### 3.3.5. Adverse Reactions

The common adverse reactions contained liver function injury, myelosuppression, gastrointestinal reactions, anemia, hypothyroidism, and reactive capillary hyperplasia. The results of heterogeneity test indicated that chi^2^ = 17.27, df = 14, *P* = 0.24, and *I*^2^ = 19%. No obvious heterogeneity was found among the contained research data. The analysis of random effect model (Figure 8) indicated that there exhibited no notable difference in the incidence of adverse reaction (*P* > 0.05). It has suggested that routine chemotherapy associated with immuno-checkpoint inhibitor therapy would not notably increase the adverse reactions of patients with advanced GC.

## 4. Analysis and Discussion

The ICIs can restore the immune response by blocking the process of immune escape. At present, immunotherapy has been successfully applied in solid cancers such as advanced head and neck squamous cell carcinoma, non-small-cell lung cancer, and malignant melanoma, and gratifying results have been obtained in the early study of GC [23]. For patients with advanced GC, two or three kinds of drugs associated with chemotherapy and targeted therapy are the main means of drug therapy at present, but long-term use of highly toxic chemotherapeutic drugs can cause drug accumulation and cause severe discomfort in patients. In clinical practice, some patients often refuse chemotherapy due to adverse reactions or other reasons, resulting in rapid tumor progression. There is limited evidence that targeted therapy can improve the prognosis of patients with GC, so it is necessary to explore new treatment models. Immunotherapy has gradually attracted medical attention. It is a landmark development in the field of immune oncology that ICIs were developed [24]. At present, the most studied ICIs are PD-1 inhibitors. Many kinds of malignant tumors have been shown to benefit from PD-1 inhibitors in terms of enhancing antitumor immunity, promoting immune-mediated tumor cell elimination, and improving overall survival rates [25]. This paper was to systematically assess the clinical effect and survival time of immune checkpoint inhibitor (ICIs) in advanced gastric cancer (GC) and adverse reactions to provide evidence-based medicine for its enhancement and adoption.

Tumor cells mainly escape the monitoring of immune response through the coinhibitory signal pathway mediated by immune checkpoint [26]. It has aroused great interest in the application of immunotherapy in patients with advanced GC, thus triggering several key clinical trials. In view of this theory, scholars began to try to develop and apply ICIs. PD-1 is the main inhibitory molecule on the surface of T cells and attaches importance to the negative regulation of immune response [27]. It has been confirmed that tumor microenvironment can induce the expression of PD-1 on tumor surface. PD-1 inhibitors, as common clinical ICIs, can induce and enhance antitumor immune response. Camrelizumab is a PD-1 inhibitor independently developed in China, which has been officially permitted by the State Drug Administration in May 2019 [28]. Cytotoxic T lymphocyte associated antigen-4 and PD-1 are the most concerned immune checkpoints. PD-1 is mainly expressed on the surface of tumor infiltrating lymphocytes, B cells, natural killer cells, and dendritic cells and binds to PD-L1, which can make activated T cells become nonreactive T cells [29, 30]. Associated with the results of this study, the disease control rate of the study group was notably better. It is suggested that the use of ICIs when treating patients with advanced GC can notably enhance the disease control rate, indicating that ICIs has obvious therapeutic effect on patients with GC. In addition, the drug can inhibit tumor progression and reduce the volume of tumor. PFS of the study group was notably longer after treatment. It is suggested that the treatment with ICIs can notably prolong the survival time of patients with advanced GC. The prolongation of survival time also reflects the exact effect of the drug, indicating that ICIs can fundamentally improve the condition of the patients. The short-term and long-term effects are reliable and can effectively prolong the survival time of patients. In tumor immunity, the immune system can recognize and get rid of tumor cells to prevent the progression of cancer. Nevertheless, tumor cells can avoid recognition and killing by immune system through immune escape, thus developing into malignant proliferation. During the period of malignant proliferation of tumor cells, they can escape immune surveillance by constantly changing the antigen phenotype and then suppress the antitumor immune response through various immunosuppression and immunosuppressive factors in the tumor microenvironment to form immune escape.

At present, clinical trials of camrelizumab when treating many kinds of tumors have been carried out. The results show that camrelizumab can increase the CR rate of relapsed/refractory classical Hodgkin's lymphoma and the objective remission rate of advanced non-small-cell lung cancer, advanced esophageal squamous cell carcinoma, and advanced GC. Clinical studies have confirmed that the immune system can enhance the immune response to tumor, to enhance the ability of autoimmune system to clear tumor cells by strengthening the inhibition of PD-1/PD-L1 pathway to achieve the purpose of antitumor. The improvement of immune function indexes in the study group was notably better after treatment. It is fully proved that immunotherapy associated with chemotherapy can improve the synergism. On the one hand, chemotherapy can obviously damage the normal cell function of the body while killing tumor cells, resulting in low immunity of patients. Immunotherapy can protect and improve the immune function of the body, reshape the antitumor immune system, enhance the antitumor effect, prolong the survival time, and improve the quality of life. Therefore, the immunity of patients has been greatly improved after the application of ICIs, which is of positive significance to the treatment and rehabilitation of the disease. Four articles in this study compared the levels of CEA and CA199 after treatment. It is suggested that the use of ICIs when treating patients with advanced GC can better inhibit tumor progression and alleviate the disease. It is considered that PD-1 inhibitors can better reduce immunosuppression, enhance antitumor immune response, and effectively prevent the progression of disease. As important tumor markers, the levels of serum CEA and CA199 can accurately reflect the disease control of patients. In this study, the levels of serum CEA and CA199 in the study group decreased notably, indicating that ICIs have a good effect on advanced GC.

No notable difference was discovered in the incidence of adverse reactions. It is suggested that routine chemotherapy associated with ICIs will not notably increase the adverse reactions of patients with advanced GC, indicating that immuno-checkpoint inhibitors are safe and suitable for patients with severe conditions. Patients are well tolerated and can be safely used. The limitations of the study are as follows: (1) the inclusion and exclusion criteria are relatively strict, and the final number of included literature is relatively small; (2) the source of heterogeneity cannot be found through subgroup analysis, which needs to be followed up by scholars, and the results of this study need to provide more support. More high-quality randomized controlled trials are needed to verify.

## 5. Conclusion

To sum up, ICIs have high clinical application value in advanced GC. Combined chemotherapy can successfully enhance the level of T lymphocytes, regulate the function of immune system, and prolong the survival time of patients. In addition, the adverse reactions are within a controllable range.

## Figures and Tables

**Figure 1:** Illustration of literature screening.

**Figure 2:** Risk of bias chart.

**Figure 3:** Summary chart of risk bias.

**Figure 4:** Forest plot of meta-analysis of disease control rate.

**Figure 5:** Forest plot of meta-analysis of levels of serum tumor markers.

**Figure 6:** Forest plot of meta-analysis of immune function index level.

**Figure 7:** Forest plot of meta-analysis of survival.

**Figure 8:** Forest plot of meta-analysis of adverse reactions.

**Table 1:** Basic characteristics of literature.

Include the literature	Year of publication	*N* (C/T)	Intervention method		Outcome index	Course of treatment	Whether it is random or not	Whether it is blind or not
			C	T				
Zheng Guili [17]	2021	40/40	FOLFOX4Chemotherapy regimen	FOLFOX4Chemotherapy regimen+PD-1Inhibitor	①②③	6 courses of treatment	Yes	No
Liang Lijun [18]	2022	43/43	Irinotecan/paclitaxel + tigio + apatinib mesylate	Irinotecan/paclitaxel + tigio + apatinib mesylate + Carrell monoclonal antibody	①④⑤	24 weeks	Yes	No
Shen Wang [19]	2022	45/43	Alotinib	Alotinib + Carrilizu monoclonal antibody	①②⑤	4 courses of treatment	Yes	No
Zhang Lianhua [20]	2021	40/40	Docetaxel + irinotecan hydrochloride + tigio	Docetaxel + irinotecan hydrochloride + tigio + Carrell monoclonal antibody	①③⑤	3 cycles	No	No
Tu Huiyang [21]	2021	38/38	XELOX/FOLFOX chemotherapy regimen	XELOX/FOLFOX chemotherapy regimen + pablizumab	①②③	3 cycles	Yes	No
Wang Junsong [22]	2022	40/42	Oxaliplatin + capecitabine	Oxaliplatin + capecitabine + Pabolizhu monoclonal antibody	①④⑤	To the progress of the disease	Yes	No

Note: C: control group; T: study group; ①: clinical efficacy; ②: immune function index; ③: tumor marker level; ④: survival time; ⑤: adverse reactions.

## Data Availability

The datasets used and analyzed during the current study are available from the corresponding author upon reasonable request.
